This article has been retracted.

# Efficacy of Human-Recombinant Epidermal Growth Factor Combined with Povidone-Iodine for Pressure Ulcers and Its Influence on Inflammatory Cytokines

**DOI:** 10.1155/2022/3878320

**Published:** 2022-08-25

**Authors:** Zunjiang Zhao, Dalun Lv, Baode Zhang, Liu Yong, Rongtao Zhang, Xiukun Wang

**Affiliations:** ^1^Department of Burns and Plastic Surgery, The First Affiliated Hospital of Wannan Medical College, Wuhu, 241004 Anhui, China; ^2^Department of Burns and Plastic Surgery, Lu'an People's Hospital, Anhui Medical University, Lu'an, 237005 Anhui, China

## Abstract

**Purpose:**

To determine the clinical efficacy of recombinant human epidermal growth factor (rh-EGF) combined with povidone-iodine (PVI) on patients with pressure ulcers (PUs).

**Methods:**

One hundred and five PU patients treated between January 2018 and January 2021 were enrolled and retrospectively analyzed. Of them, 50 patients who received conventional treatment were assigned to the control group (Con group), while 55 patients treated with rh-EGF combined with PVI were assigned to the observation group (Obs group). The two groups were compared in clinical efficacy, PU alleviation (total area reduction rate, total depth reduction rate, and total volume reduction rate), healing time, pain degree (Visual Analog Scale [VAS] score), inflammatory indexes (interleukin-8 [IL-8], tumor necrosis factor-*α* [TNF-*α*], and hypersensitive C reactive protein [hs-CRP]), and hydroxyproline content in the wound.

**Results:**

The Obs group yielded a higher total effective rate than the Con group (*P* < 0.05). The Obs group also experienced statistically shorter healing time and milder pain, with better PU alleviation and lower levels of inflammation indexes compared with the Con group (all *P* < 0.05). In addition, a higher hydroxyproline content in the wound was found in the Obs group.

**Conclusions:**

All in all, rh-EGF combined with PVI has a definite curative effect on patients with PUs. It can promote PU alleviation and hydroxyproline secretion in the wound and inhibit pain and inflammatory reactions, which is worthy of clinical promotion.

## 1. Introduction

Pressure ulcers (PUs) are a kind of an unbearable surgical disease, often accompanied by high medical costs [1, 2]. Patients with PUs will have serious pain and may even face a life-threatening infection [3]. PUs are attributed to ischemia and hypoxia after local tissue is under pressure, triggering tissue necrosis and inflammatory reaction [4]. According to epidemiological statistics, over 3.1 million adults are afflicted by PUs worldwide every year, with a resulting risk of death that is 2-6 times that of other patients [5]. Accordingly, optimizing the treatment strategy of PUs to provide patients with more suitable and ideal treatment options is of great practical significance for curbing patients' illness and relieving pain.

Recent research shows that a growing number of novel technologies, such as recombinant human epidermal growth factor (rh-EGF) and povidone iodine (PVI), contribute to accelerated wound healing [6, 7]. EGF is shown to promote skin repair and remodeling by stimulating the growth of epithelial cells in wounds, thus speeding up wound healing [8, 9]. In previous studies [10–12], rh-EGF was applied to the treatment of diabetic foot ulcer, burn wound, and cesarean section-caused wound scar, and a certain effectiveness, safety, and high wound healing rate were demonstrated, while PVI is an iodophor-based antibacterial agent with a variety of properties, including the ability to penetrate biofilm, anti-inflammatory effects, low cytotoxicity, and good tolerance, which is conducive to wound healing [13]. Evidence has indicated that PVI facilitates wound healing by promoting *α*-SMA and TGF-*β* secretion, neovascularization and re-epithelialization [14]. According to research related to animals [15], low concentration of PVI ointment can not only strongly accelerate the wound healing of earlobe ulcers in rabbits, and also effectively promote the wound healing of full-thickness skin ulcers and reduce the wound size and inflammation in rats.

At the present stage, research on the application of rh-EGF combined with PVI in the treatment of PUs is scant. Accordingly, this study probed into their combination in terms of efficacy, PU alleviation, healing time, pain degree, and inflammation, aiming at filling the gaps in this area and providing clinical reference and new opportunities for the treatment of PU patients.

## 2. Materials and Methods

### 2.1. General Materials

One hundred and five PU patients treated between January 2018 and January 2021 were enrolled and retrospectively analyzed. Of them, 50 patients who received conventional treatment were assigned to the control group (Con group), while 55 patients treated with rh-EGF combined with PVI were assigned to the observation group (Obs group). The Con group was comprised of 24 males and 26 females, with a mean age of 64.64 ± 9.68 years, and the Obs group was comprised of 26 males and 29 females, with a mean age of 67.22 ± 10.61 years. All participants provided a signed informed consent form after being informed of the purpose of the study, and the study was conducted in strict compliance with the Declaration of Helsinki, with approval obtained from the Ethics Committee of The First Affiliated Hospital of Wannan Medical College.

### 2.2. Inclusion and Exclusion Criteria

The inclusion criteria are as follows: patients confirmed with PUs; patients with high compliance; patients able to receive the whole treatment; patients with normal cognitive ability and communication ability; and those with no infectious diseases.

The exclusion criteria are as follows: patients whose wound was cancerous; patients allergic to drugs used in this study; patients with skin ulcers caused by other causes; patients who had received other drug therapy; patients complicated with other severe diseases; patients with blood system diseases; patients with diabetes mellitus; and pregnant and lactating women.

### 2.3. Therapy Means

For the Con group, the wound was cleaned with normal saline to remove blisters, ulcers, and/or necrotic tissues and then irradiated with infrared lamp for 30 min, followed by cleaning and disinfection. Then, wet compressing with gentamicin wet gauze was performed, after which the wound was covered and bandaged with sterile dressing. The dressing was changed 1-2 times a day until the wound healed.

For the Obs group, the wound was treated by cleaning, disinfection, and infrared irradiation in the same way, followed by the application of 10% PVI cream (Shen Zhen Haisi'an Biotechnology Co., Ltd., 30101477) for 10 min. Subsequently, the wound was cleaned again, followed by even application of rh-EGF gel (Shanghai Jingfeng Biotechnology Co., Ltd., TF-2049P) that was made to fully contact the wound. Before dressing, the wound was covered with gauze containing 10% PVI cream and then covered and wrapped with sterile dressings. Dressing was changed once a day until the wound healed.

### 2.4. Outcome Measures

#### 2.4.1. Clinical Efficacy

Cured: the wound healed, scabbed, and shed; markedly effective: the wound surface was obviously reduced, with significant pain relief and no secretion; effective: the wound surface was reduced, with less secretion, and the pain was alleviated; ineffective: none of the above criteria were met. The total effective rate = (the number of cured patients + remarkably effectively treated patients + effectively treated patients)/the total number of patients × 100%.

#### 2.4.2. PU Alleviation

PU alleviation was evaluated from the total area reduction rate, total depth reduction rate, and total volume reduction rate based on a paper digital ruler.

#### 2.4.3. Healing Time

The time of complete wound healing, escharosis, and shedding was recorded.

#### 2.4.4. Pain Degree

With a total score of 0-10 points, the Visual Analog Scale (VAS) was adopted for pain degree evaluation before therapy and 7 days after therapy [16]. A higher score indicates more severe pain.

#### 2.4.5. Inflammation Indexes

Before and 7 days after therapy, serum of each participant was collected, followed by determination of inflammatory indexes by enzyme-linked immunosorbent assay (ELISA) with human interleukin-8 (IL-8), tumor necrosis factor-*α* (TNF-*α*), and hypersensitive C reactive protein (hs-CRP) ELISA kits (Wuhan Yipu Biotechnology Co., Ltd., YX-E10139, YX-E10110, and YX-E111) under strict kit instructions [17].

#### 2.4.6. Hydroxyproline Content in the Wound

After 7 days of treatment, a small piece of wound tissue of each patient was collected to determine hydroxyproline content by the alkali hydrolysis colorimetry with a hydroxyproline kit (Beijing Biolab Technology Co., Ltd., KFS357).

In this study, clinical efficacy, pain degree, inflammatory indicators and wound hydroxyproline content were the primary outcomes measures, while PU alleviation and healing time were secondary measures.

### 2.5. Statistical Analyses

GraphPad Prism 6 (GraphPad Software, San Diego, USA) was adopted for data analyses and figure plotting. Counting data (gender, age, wound site, medical history of PUs, etc.) denoted by cases/percentage (n/%)) were compared via the chi-square test between groups. Intergroup comparison of measurement data (average age, wound area, total area reduction rate, total depth reduction rate, total volume reduction rate, etc.) represented by mean ± SEM was conducted by the independent-samples *t*-test, and intro-group comparison of them before and after therapy was conducted via the paired *t*-test. *P* < 0.05 denotes a remarkable difference.

## 3. Results

### 3.1. Baseline Data

No statistical differences were observed between the two groups in gender, age, average age, wound area, wound site, medical history of PUs, education level, drinking history, place of residence, and marital status (all *P* > 0.05, Table 1).

### 3.2. Clinical Efficacy

The Obs group yielded a statistically higher total effective rate than the Con group (*P* < 0.05, Table 2).

### 3.3. PU Alleviation in the Two Groups

The Obs group showed statistically higher rates of total area reduction, total depth reduction, and total volume reduction than the Con group (all *P* < 0.05, Figure 1).

### 3.4. Healing Time and Pain Degree of the Two Groups

The Obs group experienced a statistically shorter healing time than the Con group (*P* < 0.05). In addition, VAS scores of the two groups were not greatly different before therapy (*P* > 0.05), but the scores of them decreased statistically after therapy, with a lower VAS score in the Obs group (*P* < 0.05) (Figure 2).

### 3.5. Inflammatory Indexes in the Two Groups

Before therapy, the two groups were not statistically different in inflammatory indexes including IL-8, TNF-*α*, and hs-CRP (all *P* > 0.05); but after therapy, the three inflammatory indexes decreased notably, with lower levels of them in the Obs group compared with the Con group (all *P* < 0.05, Figure 3).

### 3.6. Hydroxyproline Content in the Wound in the Two Groups

After 3 days of therapy, the hydroxyproline content in the wound between the two groups was not statistically different (*P* > 0.05). After 6 days and 9 days of therapy, the hydroxyproline content in the wound in the two groups was notably higher than that after 3 days of therapy and was statistically higher in the Obs group compared with the Con group (both *P* < 0.05, Figure 4).

## 4. Discussion

PUs, a chronic skin disease, refer to lesions or injuries of the underlying tissues of the skin mainly triggered by pressure, shear force, and friction [18]. Its pathogenesis involves physiological processes such as ischemia-reperfusion injury, poor lymphatic drainage, cell deformation, and excessive apoptosis, which eventually lead to chronic inflammation and healing disorders [19]. rh-EGF and PVI are both topical drugs that are conducive to wound healing [20]. This study mainly evaluated the clinical advantages of the combination of rh-EGF and PVI in PUs compared with conventional drugs.

Many researchers have carried out relevant studies on topical drugs for the treatment of PUs. For example, Niu [21] conducted research on the application of Mayinglong Shexiang Hemorrhoids Cream combined with Pearl Powder in the treatment of severe PUs, and the results showed that this therapy could not only significantly reduce wound pain, but also effectively lower the risk of complications. Kucan et al. [22] reported that Silver Sulfadiazine Cream has excellent clinical effect in the treatment of chronic PUs, which can significantly reduce the amount of bacteria on the wound tissue of patients in a relatively short time. And Zolfagharnezhad et al. [23] pointed out that the healing process of stage I or stage II PUs in severe patients can be significantly improved under the intervention of 3% nifedipine ointment. In our study, the Obs group was treated with rh-EGF + PVI, while the Con group was treated with conventional medication. In terms of efficacy evaluation, the Obs group showed a statistically higher total effective rate than the Con group (96.36% *vs.* 84.00%), suggesting the positive effects of rh-EGF combined with PVI on the improvement of efficacy. According to previous research, EGF can accelerate wound healing by promoting granulation tissue formation, and its mechanism is closely associated with the activation of EGF on the behaviors of fibroblasts [24, 25]. With anti-inflammatory and analgesic effects, PVI can strongly accelerate granulation growth of wound surface [26, 27], while the combination of Rh-EGF and PV, with higher efficacy on PUs, facilitates the granulation growth of wound surface. We also analyzed and compared PU alleviation between the two groups from total area reduction rate, total depth reduction rate, and total volume reduction rate. The Obs group showed a better PU alleviation than the Con group. In addition, the Obs group experienced a significantly shorter healing time and milder pain than the Con group. The above results suggest the ability of the combined medication in substantially improving the wound condition and the growth of granulation tissue and reducing the discomfort induced by the disease. We also evaluated inflammatory indexes of the two groups. As is known to all, excessive secretion of inflammatory factors including IL-8, TNF-*α*, and hs-CRP will hinder wound healing, and inhibiting these inflammatory factors can prevent the inflammatory cascade reaction and promote wound healing [28, 29]. In our study, inflammatory indexes (IL-8, TNF-*α*, and hs-CRP) in the Obs group were significantly inhibited after the combined treatment and were all lower than those in the Con group, suggesting favorable inhibitory effects of the combination of drugs on inflammatory factors. Moreover, the Obs group showed a notably higher amount of hydroxyproline secretion in the wound with the passage of time. The increase of hydroxyproline can promote collagen synthesis during skin wound repair [30]. It follows from the above that the combined medication can increase hydroxyproline secretion in the wound, which in turn promotes collagen synthesis to accelerate wound healing.

This study has confirmed the remarkable clinical effect of rh-EGF combined with PVI in the treatment of PU patients, but it still has some limitations. First, we can supplement the mechanism of rh-EGF combined with PVI in cell models from the molecular perspective to further understand the mechanism of the action on wound healing process. Second, the quality of life of patient after treatment can be supplemented to analyze the influence of the two treatment methods on patients' quality of life. Finally, we can increase the sample size to improve the accuracy of the experimental results. In addition, this study is novel in the following aspects. First, the clinical efficacy of rh-EGF combined with PVI in the treatment of PU and the recovery degree of wound healing were confirmed from the aspects of clinical efficacy and PU alleviation. Second, from the perspectives of healing time and pain degree, it was determined that the combined treatment has beneficial effects on the recovery speed and pain relief of patients. The third is to analyze the underlying mechanism of the combined treatment from inflammatory indexes and hydroxyproline content in the wound. It was found that rh-EGF combined with PVI may promote wound healing by inhibiting the inflammatory response and promoting hydroxyproline release on the wound surface, thus achieving the purpose of treating PUs.

## 5. Conclusion

To sum up, rh-EGF combined with PVI can significantly improve the clinical efficacy of PU patients by alleviating PUs, promoting wound healing, and reducing pain and inflammation, which can be a new treatment option for PU patients.

## Figures and Tables

**Figure 1:** PU alleviation in the two groups. (a) The observation group showed a statistically higher total area reduction rate than the control group. (b) The observation group showed a statistically higher total depth reduction rate than the control group. (c) The observation group showed a statistically higher total volume reduction rate than the control group. Note: ^∗^*P* < 0.05; ^∗∗^*P* < 0.01.

**Figure 2:** Healing time and pain degree of the two groups. (a) The observation group experienced statistically shorter healing time than the control group. (b) The observation group experienced statistically milder pain degree than the control group. Notes: ^∗^*P* < 0.05; ^∗∗^*P* < 0.01.

**Figure 3:** Inflammation indexes in the two groups. (a) After therapy, IL-8 in the observation group decreased statistically, which was lower than that in the control group. (b) After therapy, TNF-*α* in the observation group decreased statistically, which was lower than that in the control group. (c) After therapy, hs-CRP in the observation group decreased statistically, which was lower than that in the control group. Notes: ^∗^*P* < 0.05; ^∗∗^*P* < 0.01.

**Figure 4:** Hydroxyproline content in the wound in the two groups. ^∗^*P* < 0.05*vs.* the level after 3 days of therapy; ^∗∗^*P* < 0.01*vs.* the level after 3 days of therapy; ^#^*P* < 0.05*vs.* the control group.

**Table 1:** Baseline data of the two groups [*n*(%), mean ± SEM].

Factors	*n*	Control group (*n* = 50)	Observation group (*n* = 55)	*χ* ^2^/*t*	*P* value
Sex				0.006	0.941
Male	50	24 (48.00)	26 (47.27)		
Female	55	26 (52.00)	29 (52.73)		
Age (Y)				0.405	0.525
<65	47	24 (48.00)	23 (41.82)		
≥65	58	26 (52.00)	32 (58.18)		
Average age (Y)	105	64.64 ± 9.68	67.22 ± 10.61	1.297	0.197
Wound area (cm^2^)	105	70.22 ± 14.04	71.72 ± 14.91	0.529	0.598
Wound site				0.542	0.462
Arms and legs	28	15 (30.00)	13 (23.64)		
Trunk	77	35 (70.00)	42 (76.36)		
Medical history of PUs				0.549	0.459
No	87	40 (80.00)	47 (85.45)		
Yes	18	10 (20.00)	8 (14.55)		
Drinking history				0.159	0.690
No	63	31 (62.00)	32 (58.18)		
Yes	42	19 (38.00)	23 (41.82)		
Place of residence				0.095	0.757
Urban area	75	35 (70.00)	40 (72.73)		
Rural area	30	15 (30.00)	15 (27.27)		
Marital status				0.350	0.554
Unmarried	64	29 (58.00)	35 (63.64)		
Married	41	21 (42.00)	20 (36.36)		

**Table 2:** Clinical efficacy on the two groups [*n*, (%)].

Group	*n*	Cured	Markedly effective	Effective	Ineffective	The total effective rate (%)
The control group	50	25 (50.00)	15 (30.00)	2 (4.00)	8 (16.00)	42 (84.00)
The observation group	55	44 (80.00)	6 (10.91)	3 (5.45)	2 (3.64)	53 (96.36)
*χ* ^2^ value	—	—	—	—	—	4.646
*P* value	—	—	—	—	—	0.031

## Data Availability

The simulation experiment data used to support the findings of this study are available from the corresponding author upon request.
